# A Critical Review of the Effect of Dietary Fiber Intake on the Prevention of Colorectal Cancer in Eastern Asian Countries

**DOI:** 10.1155/2021/6680698

**Published:** 2021-01-16

**Authors:** Yunfan Yang, Li Yang, Liping Zhou, Siyuan Tang

**Affiliations:** ^1^Changde Vocational Technical College, Changde, Hunan, China; ^2^Xiangya School of Nursing, Central South University, Changsha, Hunan, China

## Abstract

**Background:**

Colorectal cancer has become the second most common type of cancer in females and the third most common type of cancer in males. The incidence rate of colorectal cancer is increasing along with the change of lifestyle and dietary habits in East Asia. The cause of colorectal cancer is complex; environmental factors and genetic factors affect each other. Dietary fiber is considered as the prevention of colorectal cancer. Epidemiological data in Europe and America have suggested that dietary fiber intake is negatively correlated with colorectal cancer incidence rate. However, the evidence among different populations is inconsistent, and little is known about these associations in Eastern Asian areas.

**Objectives:**

To critically review all available human epidemiological data on the relationship between dietary fiber intake and colorectal cancer in Eastern Asian countries and make recommendations for these populations. *Methodology*. PubMed and Embase were used to search online research papers regarding the relationship between dietary fiber intake and the risk of colorectal cancer in Eastern Asian. We located 9 publications, of which the sample size ranged from 266 to 78, 326.

**Results:**

Five case-control studies, as well as one prospective study, have examined significant preventive effects of dietary fiber intake on the risk of colorectal cancer while evidence from three prospective cohorts suggested no preventive effects of dietary fiber intake on colorectal cancer among these populations. There is no consistent conclusion on the protective effect of dietary fiber from different sources and types.

**Conclusion:**

The association between dietary fiber intake and colorectal cancer risk in Chinese, Japanese, and Korean is considered to be plausible by the available literature. This current review cannot substantiate the preventive effect of dietary fiber intake on colorectal cancer due to the limited available evidence analyzed.

## 1. Introduction

### 1.1. Dietary Fiber

Dietary fiber is one of the essential nutrients for maintaining human health and is only obtained from plant foods, for example, vegetables, fruits, soy, and cereals [1]. Dietary fiber is a type of carbohydrate which is undigested and nonabsorbed in the small intestine but can be fermented in the large intestine [2]. They are mainly categorized as soluble fibers and insoluble fibers. Almost all plant foods, for example, beans and vegetables, contain both soluble and insoluble fibers but vary in the proportion of each kind of fiber [1]. Dietary fiber has many benefits to prevent various diseases such as heart disease, type 2 diabetes, digestive diseases, and some cancers [3].

### 1.2. Colorectal Cancer

Colorectal cancer has become the second most common type of cancer in females and the third most common type of cancer in males [4]. In 2008, colorectal cancer contributed to approximately 608,700 deaths and involved more than 1.2 million new cases worldwide [4]. The speedy rise of colorectal cancer incidence has occurred among some populations historically at low risk such as Eastern Asian [4]. Therefore, there is a need to explore the risk factors of colorectal cancer among these populations, thereby lowering their incidence of colorectal cancer.

### 1.3. Colorectal Cancer and Dietary Fiber Intake

Some risk factors associated with colorectal cancer are nonmodifiable factors, for example, age [5], ethnicity [6], gender [7], and menopause [8]. However, various modifiable factors improving the risk of colorectal cancer include overweight or obesity, low level of physical activity, high intake of alcohol, and smoking [4].

Dietary habits are another risk factor in the incidence of colorectal cancer [9]. However, only the effects of red meat intake on colorectal cancer risk are consistent [10]; the effects of other nutrients like dietary fiber intake on colorectal cancer may be inconsistent [11–13].

Since epidemiologic studies have not substantiated the preventive effects of dietary fiber intake on colorectal cancer risk [14], further studies and discussions to explore the true effects of dietary fiber will be conducted. However, a majority of the epidemiological evidence was derived from non-Asian populations, and there was limited research investigating the relationship in Eastern Asian.

Therefore, the aim of this paper is to critically review original papers of case-control and cohort studies that examined the association in Eastern Asian countries (including Chinese, Japanese, and Korean) between dietary fiber intake and the risk of developing colorectal cancer and make recommendations for these populations.

## 2. Materials and Methods

PubMed and Embase were used to search online research papers regarding the relationship between dietary fiber intake and the risk of colorectal cancer in Eastern Asian. The search terms “fiber intake” or “dietary fiber” or “roughage” or “white bran” were added with “colorectal cancer” or “colorectal cancer” or “colorectal neoplasm”, in conjunction with “Chinese” or “China” or “Japanese” or “Japan” or “Korea” or “Korean”. Original papers of case-control and cohort studies only were included in the review. Titles and abstracts of studies were read and considered relevant only if an association between dietary fiber intake and colorectal cancer incidence was analyzed. In contrast, animal research and research that focused on the dietary treatment of colorectal cancer survivors or analyzed the proposed anticarcinogenic mechanisms of dietary fiber were excluded. Additionally, available research papers written in English and published since 2000 were considered as the inclusion criteria.

## 3. Results

Although relatively limited research made investigation among Eastern Asian populations, the search strategy generated 295 results. Nine out of the 14 studies identified, four prospective cohorts, and five case-control studies were selected to be analyzed, as shown in Figure 1. Nine studies were examined critically, and their findings are summarized in Table 1.

Four prospective cohort studies examined the association between total fiber intake and colorectal cancer. Three studies concluded that there was no association between dietary fiber and colorectal cancer incidence [15–17]. However, a study found that the total dietary fiber intake was associated with reduced colorectal cancer risk while soluble and insoluble dietary fiber intake had no prevention of colorectal cancer [18].

5 case-control studies reviewed analyzed the association between dietary fiber intake and colorectal cancer. Fiber intake was divided into different sources to assess, including total fiber, dietary fiber, vegetable and fruit fiber, and cereal fiber. 2 studies found that, compared to the reference category, the highest total fiber intake was associated with a significantly reduced risk of colorectal cancer [19, 21]. In addition, 2 studies, as shown in Table 1, found a significant association between high dietary fiber intake and low colorectal cancer [9, 22]. 3 studies found a significantly decreased risk of colorectal cancer in the highest vegetable and fruit fiber intake categories compared to the reference categories [19–21]. One study found a high intake of cereal fiber associated with a low risk of colorectal cancer [19]. Relative risks of colorectal cancer comparing the highest amount with the lowest amount of dietary fiber intake among nine papers were shown in Figure 2.

## 4. Discussion

### 4.1. Evidence from Prospective Cohort Studies

Shin et al. [15] conducted a prospective cohort of Chinese women for investigating the preventive effects of fiber intake on colorectal cancer risk [15]. A validated food frequency questionnaire (FFQ) including 77 food items and the Chinese Food Composition Table were applied as a measure of the daily dietary intake of fiber at the baseline survey. The data observed in the study indicates that colorectal cancer cases incline toward the elderly, postmenopausal, and low educated population, independent of the intake of vegetables and fruits. Comparing the highest quintile with the lowest quintile, the relative risk for dietary fiber intake was 1.10 (95% CI: 0.6–1.8) after adjustment for some confounding factors including folate, red meat, and milk consumption. This suggests that there is no statistically significant association between dietary fiber intake and colorectal cancer risk.

The null association between total intake of dietary fiber and the risk of colorectal cancer was consistent with previous cohort studies of American women [23, 24]. A study examining 13 prospective cohorts also failed to provide evidence for inverse associations between dietary fiber intake and colorectal cancer risk after adjustment for confounders [25]. However, evidence from the prospective investigation among European into cancer and nutrition (EPIC) studies found that dietary fiber intakes were preventive to the risk of colorectal cancer after multivariable adjustment [26, 27]. Therein, a study published in 2003 suggested a 42% (95% CI: 0.41–0.85) lower risk for colorectal cancer with doubling dietary fiber intake in calibrated models, while another found that there was a statistically significant 13% (95% CI: 0.79–0.96, per 10 g/day increase in fiber intake) reduction in the risk of colorectal cancer.

The study was well designed based on the large participants and the completed follow-up. Alternatively, the study was a prospective cohort, and differential recall bias was more likely to be eliminated than if the study had been cross-sectional as the validity of the FFQ was evaluated by comparing it with 24-hour dietary recall in the study. However, the 5.74-year median follow-up period was limited, which may result in the null result. Although a large sample could increase the external validity of the results, the population of the study only focused on Chinese women aged over 40; therefore, the results from Shin et al. [15] may not be generalizable to a wider population, especially since there was a big distinction in dietary patterns and lifestyles among different populations [9]. Furthermore, random errors in the assessment of fiber intake and potential uncontrolled confounding factors may exist in the study due to the nature of observational studies, which could limit the true relationship between dietary fiber intake and colorectal cancer risk.

Further evidence agrees with the notion that dietary fiber consumption cannot prevent colorectal cancer [16]. In a population-based prospective cohort, 61,321 Singapore Chinese were involved during a 9.8-year follow-up. The study used two patterns of dietary: meat–dim sum and vegetable–fruit–soy. Dietary fiber intake was measured using a validated 165-item FFQ. This could help to comprehensively collect dietary data, thereby improving the internal validity of the study. In the analysis, weak evidence was found for the preventive effects of dietary patterns on colorectal cancer. The findings indicated that there was no relationship between dietary fiber intake and colorectal cancer risk, although the follow-up period of the study was longer than that in other studies [15, 17]. With the prospective design, the authors suggested that the differential dietary recall had a low possibility of biasing the results. However, the analysis lacked standardization for assessing dietary patterns. This could reduce the accuracy of dietary data and therefore affect the true relationship between dietary fiber intake and colorectal cancer risk.

Another study to suggest no association between dietary fiber intake and colorectal cancer risk is the Japan Public Health Centre-based Prospective Study (JPHC Study) involving 78,326 Japanese males and females during a 5.8-year follow-up [17]. The study used a validated FFQ including 138 food items, the Japanese food composition table, and the Association of Analytical Communities (AOAC) method to assess dietary fiber. The study found no statistically significant relationship between intake of dietary fiber and the risk of colorectal cancer between both males (HR = 0.85, 95% CI:0.53–1.4) and females (HR = 0.58 95% CI: 0.31–1.1), although there was little consumption of dietary fiber (the lowest quintile mean, 8.3 g/day) in relation to the increased risk of colorectal cancer in females. These findings suggested weak evidence for a preventive effect proposed for dietary fiber intake on colorectal cancer. The findings of the study also agree with those of some previous prospective studies [24, 28].

The prospective study design, a comprehensive FFQ used, and a large sample size make this a well-designed study. Potential confounding factors were considered as covariates in the analysis to reduce the effect of confounders. Additionally, the FFQ was completed before the colorectal cancer diagnosis, improving the accuracy of the data collected from dietary intake measurements, thereby minimizing the exposure recall bias. Although the study adjusted for various confounders in the analysis, the potential measure errors of dietary fiber consumption may not be totally eliminated, which may affect the results for an association between dietary fiber intake with colorectal cancer risk.

A study published one year later, however, did not report the same. They conducted the Japan Collaborative Cohort Study (JCCS) of 43,115 males and females combined; a significant inverse association was found between total dietary fiber intake and colorectal cancer risk, mainly for colon cancer [18]. These findings of the study also indicated that there was no significant difference in the decrease in colorectal cancer risk between soluble and insoluble dietary fiber intakes, as shown in Table 1. The authors explained that the high correlation between the two types of dietary fiber intake might limit the analysis on the effects of soluble and insoluble fiber, respectively. However, compared to soluble fiber, case-control studies found that insoluble fiber was strongly associated with colorectal cancer risk [9, 29].

With the prospective design and large sample size, the analysis improved the external validity of the results. In addition, recall bias was minimized by careful assessment of dietary intake. However, there was a risk of the underestimation of dietary fiber intake due to the lower number of FFQ items than that of other studies [15, 16]. This 40-item FFQ also limited the assessment of dietary fiber intake from other sources such as whole grains. Additionally, the analysis did not carefully measure other confounders such as level of physical activity and cannot exclude possible residual confounding factors. These could affect the internal validity of the results such as dietary fiber intake, suggesting that the confounders may not have been accurately measured. Applying comprehensive and objective dietary instruments would help to solve these problems.

### 4.2. Evidence from Case-Control Studies

The five case-control studies in this review incline to support the notion that there are preventive effects of dietary fiber intake on colorectal cancer. In the first research, 507 patients diagnosed with colorectal cancer (cases) and 2,535 outpatients excluding cancer (controls) in Japan were recruited as subjects [9]. The Hospital-based Epidemiologic Research Program at Aichi Cancer Center (HERPACC) questionnaire and a validated 47-item FFQ were used to estimate dietary fiber intake. The authors suggested that the changes in diet and lifestyle might explain the rising incidence of colorectal cancer among Japanese. The study adjusted for a number of confounders and found that the higher insoluble dietary fiber intake could lead to lower full adjusted odds ratios (ORs) for colon cancer (*p*=0.027). An inverse relationship was also reported between colon cancer risk and total dietary fiber intake, specifically insoluble dietary fiber. Moreover, the preventive effect of dietary fiber consumption was mainly found on colon cancer instead of rectal cancer. This may be explained through the characteristics of the rectal that it is empty most of the time, weakening the proposed preventive effects of dietary fiber [26].

The study was well designed with a number of limitations in that there was a discrepancy in the source population between cases and controls. Additionally, the study was hospital-based case-control. These may increase the risk of selection bias and recall bias, being a threat to the study validity since subjects may not be representative of the wider population and data of dietary fiber was collected retrospectively. The results of the analysis are important; since the effects of the two types of dietary fiber were explored, they also detected the protective factors and dietary risk of both colon and rectal cancer.

Three studies that followed up the Chinese population for 1 to 5 years showed that increasing dietary fiber had a significant protective effect on colorectal cancer. Zhong et al. [19] explored the association between dietary fiber intake, fiber fraction, and the risk of colorectal cancer in Chinese adults [19]. In the study, there were 613 cases with colorectal cancer and 613 matched controls including hospital-derived controls and community-derived controls. Similar to Shin et al. [15], the consumption of total dietary fiber as well as specific fiber fractions, such as vegetable fiber, fruit fiber, cereal fiber, and soy fiber, was estimated using the validated 81-item FFQ and Chinese Food Composition Table [15]. After adjusting for multiple confounding variables, 62% (95% CI: 0.27–0.55) reduced colorectal cancer risk which was related to the highest quartile intake of total dietary fiber compared to the lowest quartile. There was also evidence for an inverse association between intake of cereal fiber, vegetable, and fruit fiber and the risk of developing colorectal cancer. Similarly, a case-control study that investigated the relationship between various nutrients and food intake and the risk of colorectal cancer among Korean aged 20–80 showed that high dietary fiber intake was significantly associated with a lower incidence of colorectal cancer (OR = 0.22, 95% CI: 0.08–0.56, *p*=0.002) [22]. However, prospective studies found that there was no preventive effect of consumption of vegetable and fruit fiber on colorectal cancer, as shown in Table 1. This discrepancy may be attributed to the different characteristics of the study subjects between Western countries and Eastern Asian countries.

In addition, weak evidence for the relationship between high soy fiber consumption and decreased colorectal cancer risk was found (OR = 1.25, 95% CI = 0.88–1.76, *p*=0.17). This finding was consistent with previous prospective studies [30, 31], but Lin et al. [23] stated an exception that high intake of soy fiber was related to a low risk of colorectal cancer among Americans [23].

Similar to a previous prospective cohort study by Shin et al. [15], the median dietary fiber intake of the study was 10.5 g/day for the controls. Unlike Shin et al. [15], in addition to dietary fiber intake, the present study did assess for specific fiber fractions. Contrary to the results of Shin et al. [15], the present study found that a lower risk of colorectal cancer was related to the high consumption of total dietary fiber, vegetable fiber, and fruit fiber in both men and women. This discrepancy in results between the two studies may be explained through distinctions in the study designs. Generally, evidence from case-control studies did support the notion that there were preventive effects of dietary fiber consumption on colorectal cancer [20, 21, 29]. In contrast, weak evidence was found in most of the subsequent cohort studies exploring the association between fiber consumption and colorectal cancer risk [24, 25]. However, a community-based case-control study conducted in Japan did not substantiate the preventive effects of dietary fiber intake on colorectal cancer [32].

The study benefited from the high respondent rate and comparability in characteristics for both cases and controls, reducing the selection bias and improving the internal validity of the results. However, self-reported measures could be the limitation of the study. This could have resulted in recall bias and socially desirable bias, thereby reducing internal validity.

## 5. Conclusion

Compared to the United States and Canada, a lower intake of red meat and higher intake of cereals may be related to the lower risk of colorectal cancer in Eastern Asian [4]. However, an aging population and greatly westernized dietary consumption and lifestyle may lead to the fast growth of colorectal cancer incidence in recent years [9].

In this review, most of the studies are well designed with a large sample size, reducing the chance of two types of error. Moreover, most studies used validated FFQ and adjusted for a variety of potential confounding factors. However, the self-reported measure of dietary fiber intake of all studies may increase the chance of recall bias and socially desirable bias. In addition, the number of food items in FFQ's ranged from 40 to 165, which demonstrates that studies may be differently sensitive to dietary fiber intake. The lack of accurate assessment of dietary fiber suggests that care should be taken to interpret the results in this review.

Limitations of this review include the limited literature and lack of experimental research on the preventive effects of dietary fiber consumption on colorectal cancer, which suggests that further research may be needed on this topic. The findings of this review were obtained from Chinese, Japanese, and Korean, which may not be representative for wider populations, especially since different populations vary in dietary habits and lifestyles. Furthermore, this review only analyzed papers published since 2000, demonstrating that there is a risk of excluding additional relevant studies.

In conclusion, the association between dietary fiber intake and colorectal cancer risk in Chinese, Japanese, and Korean is considered to be plausible by the available literature. All case-control studies included as well as one prospective study have examined the significant preventive effects of dietary fiber intake on the risk of colorectal cancer in these populations, and evidence from three prospective cohorts suggested no preventive effects of dietary fiber consumption on colorectal cancer. There is no consistent finding of the protective effect of dietary fiber from different sources and types. Therefore, this current review cannot substantiate the preventive effect of dietary fiber intake on colorectal cancer due to the limited available evidence analyzed. Further prospective cohort and case-control studies among Eastern Asian populations examining the hypothesis that high dietary fiber intake is related to low risk of colorectal cancer are needed.

## Figures and Tables

**Figure 1:** Flow diagram of the systematic search of the literature on dietary fiber intake and the risk of colorectal cancer.

**Figure 2:** Relative risks of colorectal cancer comparing the highest amount with the lowest amount of dietary fiber intake.

**Table 1:** Summary of six studies on the association between dietary fiber intake and colorectal cancer risk in Chinese, Japanese, and Korea.

Author (year)	Study design	Sample characteristics	Measurements of dietary fiber	Exposure and relative risk (95% CI)	Adjustment for confounders	Findings	Study limitations
Shin et al. [15]	Prospective cohort (5.74 –year follow-up).	73, 314 Chinese women, age 40–70, 283 cases.	Validated 77-item FFQ.	Dietary fiber, 1.10 (0.6–1.8).	Age, menopausal status, education, smoking, alcohol, exercise, family history of colorectal cancer, energy, vitamin supplements.	Dietary fiber intakes did not prevent colorectal cancer.	Limited follow-up, self-reported measure, no comprehensive assessment of dietary fiber intake.

Butler et al. [16]	Prospective cohort (9.6 –year follow-up).	61, 321 Chinese men and women, age 45–74, 961 cases.	Validated 165-item FFQ.	Dietary fiber, 0.98 (0.81–1.19).	Age, gender, dialect group, interview year, diabetes mellitus, smoking, body mass index, alcohol, education, physical activity, family history of colorectal cancer, energy.	Dietary fiber intakes did not prevent colorectal cancer.	Self-reported measure, no standardization for assessment of dietary fiber intake.

Otani et al. [17]	Prospective cohort (5.8 –year follow-up).	78, 326 Japanese men and women, age 40–59 (cohort 1) and 40–69 (cohort 2), 522 cases.	Validated 138-item FFQ, AOAC method.	Dietary fiber-men, 0.85 (0.53–1.4)-women, 0.58 (0.31–1.1).	Age, alcohol, smoking, body mass index, physical exercise, folate, calcium, vitamin *D*, red meat, study area, energy.	Dietary fiber intakes did not prevent colorectal cancer.	Limited follow-up, self-reported measure, no data combined men and women.

Wakai et al. [18]	Prospective cohort (7.6 –year follow-up).	43, 115 Japanese men and women, age 40–79, 443 cases.	Validated 40-item FFQ, AOAC method.	-Total dietary fiber, 0.73 (0.51–1.03)-soluble dietary fiber, 0.69 (0.36–1.32)-insoluble dietary fiber, 1.02 (0.54–1.94).	Age, gender, area, education, family history of colorectal cancer, alcohol, smoking, body mass index, walking, exercise, sedentary work, beef/pork, energy, folate, calcium, vitamin *D*.	An inverse association between total dietary fiber intake and colorectal cancer risk, no difference in the decreased risk for colorectal cancer between soluble and insoluble dietary fiber intakes.	Self-reported measure, limited food items included in the FFQ, no careful measure for confounders.

Wakai et al. [9]	Case-control study (3–year follow-up).	507cases and 2,535 controls, Japanese, age 20–79.	Validated 47-item FFQ.	-Total dietary fiber, 0.72 (0.49–1.05)-soluble dietary fiber, 0.75 (0.52–1.10)-insoluble dietary fiber, 0.65 (0.45–0.96).	Gender, age, and year of the first visit. Season of the first visit to the hospital, the reason for the visit, family history of colorectal cancer, body mass index, exercise, alcohol drinking, smoking, multivitamin use, and energy intake.	High intakes of dietary fiber associated with low colon cancer risk, specifically insoluble dietary fiber.	Self-reported measure, limited food items included in the FFQ, a discrepancy in the source population between cases and controls.

Zhong et al. [19]	Case-control study (2–year follow-up).	613 cases and 613 controls, Chinese, age 30–75.	Validated 81-item FFQ.	-Total dietary fiber, 0.38 (0.27–0.55)-vegetable fiber, 0.45 (0.32–0.64)-fruit fiber, 0.41 (0.28–0.58),-cereal fiber, 0.48 (0.35–0.67)-soy fiber, 1.25 (0.88–1.76).	Marital status, education, regular smoking, passive smoking, leisure-time physical activity, first degree relative with cancer, total energy intake, and total animal food intake.	High intakes of total fiber, cereal fiber, vegetable fiber, and fruit fiber associated with the low risk of colorectal cancer.	Self-reported measure, different sources of controls.

Chiu et al. [20]	Case-control study (5-year follow-up).	931 cases and 1552 controls, Chinese, age 30–74.	Validated 86-item FFQ.	Fruits and vegetables-men 0.7 (0.5–1.0),-women 0.6 (0.4–0.9).	Age, total energy intake, education, body mass index, monthly family per capita income, and occupational physical activity.	High fruit and vegetable fiber intake reduces the risk of colorectal cancer.	Self-reported measure, no data combined men and women, little effect of the further adjustment in the final model, random misclassification of diet in the questionnaire.

Song et al. [21].	Case-control study (1-year follow-up).	265 cases and 252 controls, Chinese, age 30–70.	Validated 121-item FFQ.	-Total fiber intake 0.44 (0.27–0.73),-vegetable fiber intake 0.51 (0.31–0.85).	Age, gender, smoking habits, drinking habits, physical activity, body mass index (BMI), and total energy.	Vegetable fiber and total fiber associated with a low risk of colorectal cancer.	Limited follow-up, lack of validated questionnaire, little control for more confounders.

Chun et al. [22]	Case-control study (1-year follow-up).	150 cases and 116 controls, Korean, age 20–80.	Validated 102-item FFQ.	Dietary fiber 0.22 (0.08–0.56).	Gender, age, economic status, educational level, smoking, alcohol drinking frequency, and leisure-time physical activity.	High dietary fiber intakes associated with a low risk of colorectal cancer.	Limited follow-up, self-reported measure, potential recall bias, possible misclassification of dietary fiber.

## Data Availability

The data used to support the findings of this study are included within the article.

## Abbreviations

CI: Confidence intervals
95% CI: 95% confidence intervals
FFQ: Food frequency questionnaire
AOAC: Association of Analytical Communities.
